The article "Biomimetic Rotary Tillage Blade Design for Reduced Torque and Energy Requirement" was published in 2021. Journal: Appl Bionics Biomech.

# Biomimetic Rotary Tillage Blade Design for Reduced Torque and Energy Requirement

**DOI:** 10.1155/2021/8573897

**Published:** 2021-09-28

**Authors:** Yuwan Yang, Jin Tong, Yuxiang Huang, Jinguang Li, Xiaohu Jiang

**Affiliations:** ^1^College of Mechanical and Electronic Engineering, Northwest A&F University, Yangling 712100, China; ^2^College of Biological and Agricultural Engineering, Jilin University, Changchun 130022, China; ^3^Key Laboratory of Bionic Engineering, Ministry of Education, Jilin University, Changchun 130022, China

## Abstract

A rotary cultivator is a primary cultivating machine in many countries. However, it is always challenged by high operating torque and power requirement. To address this issue, biomimetic rotary tillage blades were designed in this study for reduced torque and energy requirement based on the geometric characteristics (GC) of five fore claws of mole rats, including the contour curves of the five claw tips (GC-1) and the structural characteristics of the multiclaw combination (GC-2). Herein, the optimal blade was selected by considering three factors: (1) the ratio (*r*) of claw width to lateral spacing, (2) the inclined angle (*θ*) of the multiclaw combination, and (3) the rotary speed (*n*) through the soil bin tests. The results showed that the order of influence of factors on torque was *n*, *r*, and *θ*; the optimal combination of factors with the minimal torque was *r* = 1.25, *θ* = 60°, and *n* = 240 rpm. Furthermore, the torque of the optimal blade (BB-1) was studied by comparing with a conventional (CB) and a reported optimal biomimetic blade (BB-2) in the soil bin at the rotary speed from 160 to 320 rpm. Results showed that BB-1 and BB-2 averagely reduced the torque by 13.99% and 3.74% compared with CB, respectively. The field experiment results also showed the excellent soil-cutting performance of BB-1 whose average torques were largely reduced by 17.00%, 16.88%, and 21.80% compared with CB at different rotary speeds, forward velocities, and tillage depths, respectively. It was found that the geometric structure of the five claws of mole rats could not only enhance the penetrating and sliding cutting performance of the cutting edge of BB-1 but also diminish the soil failure wedge for minimizing soil shear resistance of BB-1. Therefore, the GC of five fore claws of mole rats could inspire the development of efficient tillage or digging tools for reducing soil resistance and energy consumption.

## 1. Introduction

The rotary cultivator is a primary cultivating machine in many countries including Bangladesh, India, Nepal, Thailand, Japan, Malaysia, the People's Republic of China, and South Korea [1–4]. It can efficiently complete the operations of soil mixing, turning, pulverizing, puddling, and leveling and thereby create good seedbeds for crop growing. However, the rotary cultivator is always challenged by the large power requirement, since it needs about 80% of the power for the interaction between the rotary tillage blade and soil, such as soil cutting and throwing [5]. Studies showed that the blade shape was an important factor affecting the power requirement [6, 7]. Then, some geometrical optimizations were proposed to reduce the torque requirement of the rotary tillage blade. For example, a saw tooth angular blade of the rotary cultivator was designed and tested in field [8]. The straight blade required the least torque, average power, peak power, specific energy, and effective specific energy at 375-500 rpm [9]. The optimal biomimetic blades based on the geometrical structure of one claw tip of mole rats required lower torque than the conventional universal blade during soil-rototilling and stubble-cutting operations [10]. In fact, drag reduction can be achieved by electron osmosis, vibration, magnetization, or bionic tillage component methods. However, many challenges remain in relation to the geometrical parameters of the rotary tillage blade. In this study, novel rotary tillage blades were designed for minimizing the power requirements.

The article "Biomimetic Rotary Tillage Blade Design for Reduced Torque and Energy Requirement" was published in 2021. Journal: Appl Bionics Biomech.

Bionic methods based on biological principles have been applied in engineering systems and modern technologies to improve or create new techniques [11, 12]. The sources of successful biomimetic designs include the excellent geometric characteristics of animals, such as the segmented body of earthworms, the nonsmooth morphology of the head of dung beetles, and the strong and sharp claws of mole rats. For example, a biomimetic bulldozer featuring the wavy body surface of earthworm was able to crush soil clods than a traditional smooth bulldozer [13]. A biomimetic rough curved soil-cutting blade based on the geometrical rough structures of soil-burrowing animals could experimentally reduce soil adhesion and friction and thereby considerably decrease the draught forces [14]. A biomimetic disc based on the profile curves of the second digit of mole fore claws performed better in structural strength and cutting efficiency using finite element analysis [15].

Mole rats are born diggers that have adapted to a strict subterranean lifestyle [16]. They possess outstanding digging performance in digging tunnels over 91 m overnight. A mole rat exerts the greatest power to the soil following the rotation of humerus around its own long axis and repeats this process [16, 17] as shown in Figure 1(a). The principle of the claw-soil interaction is similar to that between the rotary tillage blade and soil as shown in Figure 1(b). In fact, the claw-soil interaction is closely related with the soil-cutting performance of animals [18]. Each of the mole hand has five fingers, which each possess a large, sharp, and powerful claw. Ji et al. [19] only characterized the geometry of the second claw of mole rats. However, when a mole rat cuts soil, the five fore claws always work synergistically with an opened-up but coplane configuration, which is described as multiclaw combination, for efficient cutting [20]. Moreover, the contour curves of the five claw tips also significantly affect the soil-cutting performance of mole rats.

The article "Biomimetic Rotary Tillage Blade Design for Reduced Torque and Energy Requirement" was published in 2021. Journal: Appl Bionics Biomech.

In this study, the geometric characteristics (GC) of the five fore claws, including the contour curves of the five claw tips (GC-1) and the structural characteristics of the multiclaw combination (GC-2) inspired us to optimize the biomimetic rotary tillage blades for efficient working. And the torque requirements of biomimetic blades were researched through soil bin tests and field experiments at different tillage conditions. The aim was to achieve an optimal biomimetic blade (BB-1) and reveal the effects of the geometric characteristics of the five fore claws on the soil-cutting performance.

## 2. Geometric Characteristics of Five Fore Claws of Mole Rats

### 2.1. Five Fore Claws of Mole Rats

Mole rats (*Scaptochirus*, *Talpidae*) (Figure 2(a)) were obtained from the northeast region of China where they are most common and inhabit mostly underground. Their broad and strong hands which consist of five different claws (see Figure 2(b)) were scanned by a three-dimensional laser scanner (Handyscan700, Creaform, Canada), and the point cloud of the five claws (see Figure 3) was created with the reverse engineering software program of ImageWare (version 13, Siemens PLM software, Germany). After a series of procedures, such as smoothing, reducing, and simplification, the five claws were reconstructed into a surface, and then, it was generated as an entity from a surface in SolidWorks software. Then, the characteristics of the contour curves of the five claw tips and the multiclaw combination were described in the following.

### 2.2. The Contour Curve Characteristics of Five Claw Tips (GC-1)

The claw tip of mole rats reduces the soil penetration resistance and makes the digging more efficient and fast. In this study, the curves of the five claw tips of mole rats were extracted in the reverse engineering software program of ImageWare (version 13, Siemens PLM software, Germany). The extracted points of the curves of the five claw tips were adjusted and plotted in the AutoCAD 2014 software for obtaining their data information. These point data information were imported to the OriginPro 9.1 software for quantitative analysis (Figure 4). The contour curves of the five claw tips were fitted based on the least square method, and the Gaussian function equations of the fitted contour curves were obtained simultaneously as shown in Equation (1). The values of the coefficient of determination (*R*^2^) were all above 0.95 showing that the fitting curves were close to the contour curves of the five claw tips. Furthermore, the sums of squares for error (SSE) were all less than 0.05 indicating that the Gaussian function equations could accurately describe the contour curve characteristics of five claw tips.

(1) $$\begin{array}{c} y=a_{1}e^{-{\left(\left(x+b_{1}\right)/c_{1}\right)}^{2}}+a_{2}e^{-{\left(\left(x+b_{2}\right)/c_{2}\right)}^{2}}, \end{array}$$

where *a*_1_, *a*_2_, *b*_1_, *b*_2_, *c*_1_, and *c*_2_ are the coefficient of the fitting equations and recorded in Table 1.

The article "Biomimetic Rotary Tillage Blade Design for Reduced Torque and Energy Requirement" was published in 2021. Journal: Appl Bionics Biomech.

### 2.3. Structural Characteristics of the Multiclaw Combination (GC-2)

The five claws differ in structural characteristics. From Figure 2(b), the 3rd claw was considerably longer than the 1st, 2nd, 4th, and 5th claws with the 5th claw being very small. The claw dimension and the lateral spacing difference between two adjacent claws are important parameters for defining the structure characteristics of multiclaw combination as shown in Figure 2(b). The length (*L*) is defined as the vertical extension of a claw. The variation of the horizontal dimension along the claw direction is typically very small, and thus, the width (*W*) is determined at the middle of the claw (*L*/2). The lateral spacing between two adjacent claws is labelled as Δ*x*. All of the parameters were recorded and presented in Table 2 according to the previous literature [20]. From the studies by Godwin [21, 22], the working depth/width ratio and the tine spacing are the important parameters to determine the categories of blades, soil failure pattern, and soil forces. Therefore, to clarify the structural and working characteristics of multiclaw combination, we defined the ratio *q* of length (*L*) to width (*W*) of each claw in Equation (2) and the ratio *r* of width (*W*) to lateral spacing (Δ*x*) in Equation (3). The values of *q* and *r* were calculated according to Equations (2) and (3) and presented in Table 2. Moreover, a mathematical model was developed to describe the structural characteristics of the multiclaw combination as shown in Equation (4).

(2) $$\begin{array}{c} q=\frac{L}{W}, \end{array}$$

(3) $$\begin{array}{c} r=\frac{\Delta x}{W}, \end{array}$$

(4) $$\begin{array}{c} w_{0}=0.5W_{1}+\Delta x_{12}+\Delta x_{23}+\Delta x_{34}+\Delta x_{45}+0.5W_{5}=0.5W_{1}+r_{12}W_{2}+r_{23}W_{3}+r_{34}W_{3}+r_{45}W_{4}+0.5W_{5}=0.5\frac{L_{1}}{q_{1}}+r_{12}\frac{L_{2}}{q_{2}}+r_{23}\frac{L_{3}}{q_{3}}+r_{34}\frac{L_{3}}{q_{3}}+r_{45}\frac{L_{4}}{q_{4}}+0.5\frac{L_{5}}{q_{5}}, \end{array}$$

where *L* is the length of the claw (mm), *W* is the width of the claw (mm), Δ*x* is the lateral spacing between adjacent claws (mm), *q* is the ratio of the length (*L*) and the width (*W*), *r* is the ratio of the width (*W*) and the lateral spacing (Δ*x*), *w*_0_ is the total width of the multiclaw combination (mm), *L*_*i*_ is the length of the *i*-th claw (mm), *W*_*i*_ is the width of the *i*-th claw (mm), *q*_*i*_ is the ratio of the length (*L*) and the width (*W*) of the *i*-th claw, *r*_*ij*_ is the ratio of the width (*W*) and the lateral spacing (Δ*x*) of the *i*-th claw and the *j*-th claw, and *j* = *i* + 1, *i* = 1, 2, 3, 4.

The article "Biomimetic Rotary Tillage Blade Design for Reduced Torque and Energy Requirement" was published in 2021. Journal: Appl Bionics Biomech.

The value of *q* ranged from 2.63 to 3.41 (Table 2), indicating the five claws belonged to narrow tines, and the value of *r* ranged from 1.12 to 1.60. Clearly, the multiclaw combination also could be regarded as a multitine combination, and the lateral space between two adjacent tines was adjustable to allow mole rats to adapt to more circumstances.

## 3. Design of Biomimetic Rotary Tillage Blades

A conventional rotary tillage blade was composed of the holder, lengthwise surface, transition surface, and scoop surface as shown in Figure 5(a). When a tillage operation is performed in the field, the lengthwise surface of blade will touch soil firstly and cut open the soil, cut off, or push aside the ground stalks and weeds; and then, the scoop surface of blade will cut soil transversely and mix, turn, pulverize, and throw the tilled soil [23]. Consequently, more energy is required by the scoop surface than the lengthwise surface during the tillage operation of blade [24]. According to the geometric characteristics of five-claw combination described above, the five claws were arranged along the scoop surface of blade for reducing the soil resistance. The first two claws, the 3rd claw, and the last two claws were located along the cutting edge, at the maximal rotary radius of the blade, and along the end of the blade, respectively. The configuration of the bionic rotary tiller blade is shown in Figure 5(b). The contour curves were magnified to fit the dimension of the corresponding claw. The values of *q* and *r* referred to that of the prototype of the multiclaw combination. And the whole width (*w*_0_) of the bionic structure was set to meet the dimension requirement of the rotary tillage blade.

The article "Biomimetic Rotary Tillage Blade Design for Reduced Torque and Energy Requirement" was published in 2021. Journal: Appl Bionics Biomech.

## 4. Soil Bin Tests

### 4.1. Test Preparation

The rotary tillage tests were conducted in an indoor soil bin (Figure 6(a)) at the Jilin University, China. The soil bin (40 m long, 3 m wide, and 0.8 m deep) was used to provide a repeatable soil condition for the experiment. The soil used for the experiments (46% sand, 33% silt, and 21% clay content) is a loamy soil which is representative of a large proportion of crop-growing regions in northeast China. The soil preparation involved adding a predetermined amount of water to reach the targeted moisture content and in the following day loosening by the rotary cultivator (1GKN-125 made by Lianyungang Weidi Machinery Co., Ltd.), leveling by a scraper blade, and compacting by a roller. Finally, the soil bed was prepared with an average soil moisture content of 18.23% d.b., a bulk density of 1957 kg m^−3^, and a soil compaction of 0.68 MPa, which was suitable for rotary tillage operation.

The test equipment consisted of a power control unit, a data collection unit, a power transmission unit, and the rotary tillage blades as shown in Figure 6(a). The power control unit mainly included the soil bin trolley, which provided the blades the forward and rotary power. The data collection unit included a torque sensor (CYB-803S, 0-±100 N m) and a computer. The power transmission unit consisted of a universal joint coupling, a gear box (1 : 1 transmission ratio), a synchronous belt wheel (1 : 1 transmission ratio), a rotary shaft, and two blade holders and transmitted the power to the blades (Figure 6(b)). In this study, the selected blade (IT245) had a working radius (*R*) of 245 mm and a width (*b*) of 60 mm, which were typical with rotary tillers. According to the mathematical model as shown in Equation (3), the whole width (*w*_0_) of the bionic structure was set to be 60 mm. The soil bin was divided into three sections for avoiding interactions between consecutive test runs (Figure 7). The section (0.8 m wide and 20 m long) was set with two transition parts at both ends and a 5 m long transition part which well met the test conditions. The 10 m long stable part remained enough for collection of the experimental data. Two rotary tillage blades were fitted at 180° out of phase by the holders. The forward speed was maintained at 3 km h^−1^ and the operating depth at 80 mm following the Government Standard of Rotary Tiller in China, the same for all sections.

### 4.2. Regression Test

Regression design could efficiently obtain the sufficient and accurate information of the response variable by selecting the values of the regression variable [6]. Box-Behnken design is a common way to combine the different factors to develop a mathematical relationship between the targets and the factors with cost-effectiveness and fewer tests [25]. In order to simplify the tests and ensure the accuracy at the same time, these tests used Box-Behnken design to select factor values, conducting the test arrangements in soil bin. Due to the adjustability of the lateral spacing between adjacent claws, *r* was varied and regarded as one influential factor affecting the working performance of the rotary tillage blade. And the inclined angle (*θ*) of the multiclaw combination, defined as the angle between the five claws and the vertical line (Figure 5(b)), also affected the soil-cutting performance of the biomimetic rotary tillage blades and was selected as an influence factor. Moreover, rotary speed (*n*) also played an important role on the working performance of rotary tiller blades [26] and was as another influence factor. Here, the ratio (*r*) of width to lateral spacing was set at an interval of 0.25 from 1.25 to 1.75, the inclined angle (*θ*) was changed from 50° to 70° at an interval of 10°, and the rotary speed (*n*) ranged from 160 to 320 rpm at an interval of 80 rpm. In total, nine bionic rotary tiller blades were designed for this study. For the experiments, all the bionic blades were wire-electrode cut, tapered, and sharpened to achieve the bionic structures (Figure 8).

The article "Biomimetic Rotary Tillage Blade Design for Reduced Torque and Energy Requirement" was published in 2021. Journal: Appl Bionics Biomech.

A mathematical relationship of torque with the three factors (*r*, *θ*, *n*) was established in the Design-Expert Software (Equation (5)). The factor-level coding was given in Table 3. The test scheme included twelve factorial points and five zero points as shown in Table 4. In order to identify the influence of the above parameters on the torque, a quadratic mathematical regression method was used to establish the regression equation between each factor and the torque. Each test was repeated three times, and the average value of the torque obtained from the data collection unit was used for result analysis.

(5) $$\begin{array}{c} T=b_{0}+b_{1}x_{1}+b_{2}x_{2}+b_{3}x_{3}+b_{4}x_{1}x_{2}+b_{5}x_{1}x_{3}+b_{6}x_{2}x_{3}+b_{7}x_{1}^{2}+b_{8}x_{2}^{2}+b_{9}x_{3}^{2}, \end{array}$$

where *T* is the torque (N-m); *x*_1_, *x*_2_, and *x*_3_ are the codes; and *b* is the coefficient of the codes.

Here, the purpose of this test was to obtain a set of optimized bionic rotary tiller blade (BB-1) parameters for reduced torque requirement and analyze the influence of each factor in the regression model on the response value. Further, a comparison of the soil-cutting performance of the optimized bionic blade (BB-1) with a conventional blade (CB) and a reported biomimetic rotary tillage blade [10] (BB-2) would be conducted in the soil bin.

The article "Biomimetic Rotary Tillage Blade Design for Reduced Torque and Energy Requirement" was published in 2021. Journal: Appl Bionics Biomech.

### 4.3. Comparative Test

The optimal biomimetic blade (BB-1) obtained from the regression test was compared with two controls in the soil bin, aiming to investigate how the torque requirement was influenced by the bionic geometric characteristics. The controls were the conventional rotary tillage blade (CB) and the optimal biomimetic rotary tillage blade (BB-2) in Ref. [10] which had three arc concave teeth equally arranged on the front cutting edge with a central angle of 60°.  Figure 9 shows the three types of the blades used in the comparative test. During the comparative test, the rotary speed changed from 160 to 320 rpm at an interval of 40 rpm, and each test was repeated three times.

## 5. Field Experiments

### 5.1. Experimental Site and Equipment

The experiments were conducted in a tested field of Jilin Agricultural University, China. The soil was a loamy soil with a bulk density of 1040 kg m^−3^ measured by the oven-drying method, a water content of 20.82% measured using a TDR-300 type Soil Moisture Meter (RGB Spectrum Equipment, USA) with 12 cm probes, and a soil compaction of 0.74 MPa measured using a SC-900 type Soil Compaction Meter (RGB Spectrum Equipment, USA) with a 1/2^″^ 00 diameter cone tip. As shown in Figure 10(a), a tractor (70.8 kw, KUBOTA-M954 made by Kubota Agricultural Machinery (Suzhou) Co., Ltd.) with a rotary tiller (1GQN-230 made by Tianjin Tractor Manufacture Co., Ltd.) moved forward to cut soil, and a sensor testing system recorded the data during the cutting process. The blades were installed in the rotary tiller to connect the blades with the tractor power take-off shaft. The torque sensor (CYB-803S, 0-±1000 N m) was placed on the tractor power take-off shaft (Figure 10(b)) so that the torque of the blades could be transmitted to sensors. The detail of the experimental methods and processes could be found in our former work [27].

### 5.2. Experimental Treatment and Data Processing

The experiments compared the torque requirements between the BB-1 and CB (IT245) operated at different rotary speeds, forward velocities, and tillage depths. According to the Government Standard of Rotary Tiller in China, the rotary speed, forward velocity, and tillage depth were, respectively, set in the ranges of 150 to 350 rpm, 1 to 5 km h^−1^, and 80 to 200 mm. A four-factor random complete block design with three replications was used, as follows:

- Factor A (blade geometry)—2 treatments: CB and BB-1
- Factor B (rotary speed)—2 treatments: 254 and 267 rpm (according to the tractor power output shaft speed)
- Factor C (forward velocity)—5 treatments: 1, 2, 3, 4, and 5 km h^−1^
- Factor D (tillage depth)—3 treatments: 80, 120, and 160 mm

Treatment Factor A was randomly followed by a random allocation of two levels of Factor B at a forward velocity of 3 km h^−1^ and a tillage depth of 120 mm, randomly followed by a random allocation of five levels of Factor C at a rotary speed of 254 rpm and a tillage depth of 120 mm, randomly followed by a random allocation of three levels of Factor D at a rotary speed of 254 rpm and a forward velocity of 3 km h^−1^. In order to eliminate the effect of the acceleration of the tractor, the data were recorded continuously after the tractor had moved 10 m. During this period of data processing, the average value of torque from three replications was used in the analysis.

The article "Biomimetic Rotary Tillage Blade Design for Reduced Torque and Energy Requirement" was published in 2021. Journal: Appl Bionics Biomech.

## 6. Results

### 6.1. Results of Soil Bin Tests

#### 6.1.1. Result Analysis of Regression Test

The orthogonal test of soil cutting by the biomimetic blades was conducted in the soil bin according to the test scheme (Table 4). The torque fluctuated from 17.26 to 25.81 N-m as the factors both varied, which expressed the importance of the optimization of the tests. The data obtained in Table 4 was processed according to Equation (5) by the least square method, and the quadratic regression model was developed as follows:

(6) $$\begin{array}{c} T=18.31+0.95x_{1}+0.19x_{2}-1.56x_{3}-0.0025x_{1}x_{2}+0.012x_{1}x_{3}-0.1x_{2}x_{3}-0.25{x_{1}}^{2}+0.24{x_{2}}^{2}+5.14{x_{3}}^{2}. \end{array}$$

The ANOVA of the regression model is shown in Table 5 to analyze and judge the reliability of the regression model. Based on the *F* distribution table, the value of *F*_0.05_(9, 7) was 3.68, which was much less than the *F* value of the above regression model. And the *P* value of this model was less than 0.05, indicating that this regression model was reliable and significant. It was also highlighted by the smaller *F* value (3.25) and larger *P* value (0.1426) of the lack of fit, showing that the lack of fit was not significant and conversely the fitting results of the quadratic regression were outstanding. Moreover, the factors of *x*_1_, *x*_2_, *x*_3_, *x*_1_*x*_1_, *x*_2_*x*_2_, and *x*_3_*x*_3_ were the significant terms to influence the model due to their larger *F* values and smaller *P* values, while the other factors of *x*_1_*x*_2_, *x*_1_*x*_3_, and *x*_2_*x*_3_ were the insignificant terms due to their smaller *F* values and larger *P* values. Therefore, the effect of each factor on the torque would be analyzed as follows.

In order to obtain a single-factor model, the other two factors were fixed at 0 levels so that the submodels of the ratio of claw width to interval, the inclined angle, and the rotary speed were

(7) $$\begin{array}{c} \left\{\begin{array}{c} T_{x_{1}}=18.31+0.95x_{1}-0.25x_{1}^{2},\\ T_{x_{2}}=18.31+0.19x_{2}+0.24x_{2}^{2},\\ T_{x_{3}}=18.31+1.56x_{3}+5.14x_{3}^{2}. \end{array}\right. \end{array}$$

The single-factor models of the above formula are derived from their respective single factors to the marginal equation of the torques of each factor at different levels:

(8) $$\begin{array}{c} \left\{\begin{array}{c} T^{\prime }x_{1}=0.95-0.5x_{1},\\ T^{\prime }x_{2}=0.19+0.48x_{2},\\ T^{\prime }x_{3}=1.56+10.28x_{3}. \end{array}\right. \end{array}$$

The regression curves of the submodels and their corresponding derivation curves of factors are as shown in Figure 11. When *x* increased from -1 to 1, the change of *x*_1_ had a positive effect on *T*_*x*_ (Figure 11(b)); so, *Tx*_1_ would increase all the time with the increasing of *x* (Figure 11(a)). When *x* > −0.5, the change of *x*_2_ started to positively effect on *T*_*x*_; inversely, when *x* < −0.5, the change of *x*_2_ had a negative effect on *T*_*x*_ (Figure 11(b)); as a result, *Tx*_2_ would get the maximum or minimum near *x* = −0.5 (Figure 11(a)). When *x* > 0, the change of *x*_3_ had a significant positive effect on *T*_*x*_; oppositely, when *x* < 0, the change of *x*_3_ had a significant negative effect on *T*_*x*_ (Figure 11(b)); thus, *Tx*_3_ would get the maximum or minimum near *x* = 0 (Figure 11(a)). *T*_*x*_ was most influenced by *x*_3_ than *x*_1_ and *x*_2_, while the impact of *x*_1_ was slightly higher than *x*_2_. When the factors were at different levels, the torque would change in different degrees. Therefore, it was necessary to optimize the geometries of the blade operating at a suitable condition for meeting a lower torque requirement.

The article "Biomimetic Rotary Tillage Blade Design for Reduced Torque and Energy Requirement" was published in 2021. Journal: Appl Bionics Biomech.

#### 6.1.2. Optimization

The torque affected by the interactions of the ratio of claw width to lateral spacing (*r*), the inclined angle (*θ*), and the rotary speed (*n*) was displayed by the response surface methodology as shown in Figure 12. The response surface diagrams intuitively reflected the variation trends of torque affected by factors. The trend of torque affected by *r* and *θ* was opposite to the trends affected by *r* and *n* and *θ* and *n*. The variation of torque affected by *r* and *θ* was small (Figure 12(a)); by contrast, with *n*, the value variation of torque was relatively large (Figures 12(b) and 12(c)), indicating the factor *n* had the most significant effect on the torque than *r* and *θ*. In Figure 12(a), the torque changed more intensely affected by *r* and *θ*, which indicated that the effect of *r* was slightly higher than *θ*. These results based on the response surface diagrams of torque were basically similar to the above results obtained from Figure 11. The torque could get the minimum value within the range of *r*, *θ*, and *n* from the comparison of Figure 12(a). Consequently, when taking (*r*, *θ*, *n*) as (1.25, 60°, 240), the torque attained the minimum value, which meant that the optimized parameters were the ratio *r* = 1.25, the inclined angle *θ* = 60°, and the rotary speed *n* = 240 rpm.

The article "Biomimetic Rotary Tillage Blade Design for Reduced Torque and Energy Requirement" was published in 2021. Journal: Appl Bionics Biomech.

#### 6.1.3. Results of Comparative Test

Figure 13 shows the comparative test results of the three rotary tillage blades affected by rotary speed. The torques of three blades showed a similar trend with the varied rotary speeds. The torque decreased as the rotary speed increased from 160 to 240 rpm because of the reduction of the bite length and a smaller volume of soil per bit. And then, the torque increased when the rotary speed increased from 240 to 360 rpm due to the soil retillage and an increasing in soil acceleration. Therefore, there was a minimal torque at the rotary speed of 240 rpm. This variation trend accorded with the results of the literature [9]. Among the three blades, the BB-1 had the lowest torque requirement in the soil tillage process. On average, the BB-1 reduced the torque requirement by 13.99% than that of the CB. And the torque requirement of the BB-2 was 3.74% less than that of the CB which was paralleled to the result of the literature [10]. It indicated that the geometric characteristics of the five fore claws of mole rats have significant effects on the torque requirement of rotary tillage blades.

### 6.2. Results of Field Experiments

A comparison of the torque requirements between the BB-1 and CB conducted in field experiments at different tillage conditions is shown in Figure 14. It could be seen that the variation trends of torque of the optimized bionic blade were similar to the trends of the conventional blade regardless of tillage conditions. When the rotary speed increased from 254 to 267 rpm, the torque significantly reduced due to the reduction of the bite length of blades which was observed in previous study [9]. As the forward velocity increased from 1 to 2 km h^−1^, the torque was also enlarged rapidly due to the increase of the soil retillage as mentioned by the literature [9], whereas the soil retillage was reduced with further increases in forward velocity from 2 to 3 km h^−1^ resulting in a decline of the torque; but the torque increased once again when the forward velocity was from 3 to 5 km h^−1^ due to the increase of the bite length of blades as suggested by Salokhe et al. [28]. Therefore, the forward velocity of 3 km h^−1^ was a more suitable operating condition for the rotary tiller blades to require a lower torque. Additionally, the tillage depth was also an outstanding effect on the torque requirement of blades. The torque increased all the time with the tillage depth varied from 80 to 150 mm due to the increase of soil volume in per bit. Overall, the optimization of rotary tiller blade in this study made no impacts on the variation trends of torque with tillage conditions.

The article "Biomimetic Rotary Tillage Blade Design for Reduced Torque and Energy Requirement" was published in 2021. Journal: Appl Bionics Biomech.

On the other hand, the optimized bionic blade always far surpassed the conventional blade in the torque requirements. It was found out that the torques of the optimized bionic blade were averagely 17.00%, 16.88%, and 21.80% lower than those of conventional blade at different rotary speeds, forward velocities, and tillage depths, respectively. It could be concluded that the soil-cutting performance of the optimized bionic blade was better than that of conventional blade due to the fact of reduced torque requirement.

In summary, these results further confirmed that the scoop surface of rotary tillage blade played an important role in the torque requirement of the whole blade so that it was necessary to optimize its geometries to achieve lower energy consumption.

## 7. Discussion

In general, when the rotary tillage blade cuts soil, the lengthwise surface, the transition surface, and the scoop surface successively touched the soil. Thus, the sliding cutting performance of the cutting edge played an important role in the soil cutting [29]. Upon the soil entrance of blade, the soil was gradually broken into small clods in conformity to the Mohr-Coulomb failure criterion [30, 31]. In each circle of this broken process, a soil wedge [32] was formed in front of the blade as shown in Figure 15(a), and the required shear force followed the Coulomb formula.

### 7.1. Effect of the Contour Curve Characteristics of the Five Claw Tips (GC-1) on the Torque of BB-1 in the Soil-Cutting Process

The reported BB-2 reduced the torque requirement by 3.91% because the three concave arcs could improve the penetration performance [10]. Similarly, BB-1 also had a better penetration performance than CB, since the cutting edge could reduce the contact area with soil when the blade touched the soil. Moreover, the contour curves of the five claw tips had an excellent sliding cutting performance. The curvatures of the five claw tips were calculated as shown in Figure 16. The curvature of the 1st claw tip showed one peak of 3.5 mm^−1^ at *x* = −0.15 mm, then declined rapidly to *x* = 0.2 mm, and continued to decrease at a lower rate from *x* = 0.2 to 1.2 mm, indicating that the 1st claw tip suffered so severe soil wear that it had a better sliding cutting performance. The curvatures of the other four claw tips each had two peaks and were small between the two peaks for each tip, indicating that the middle part between the two peaks for each tip mainly cut soil, especially for the 2nd claw tip. For the 3rd claw tip, the narrow middle part between the two peaks contributed to a better penetration performance. Interestingly, the peaks of the curvatures decreased from the 1st to the 3rd claw and then increased to the 5th claw. The smaller peak of the curvature in the 3rd claw tip could avoid quick wear by soil when it penetrated into soil. On the whole, the contour curves of the five claw tips had a better penetration and sliding cutting performance. As a result, the sliding cutting action was performed at a small dip angle to reduce friction force and insure emergence from the soil, which was similar to the slide cutting performance of the fore claw of *Cryptotympana atrata nymph* [33]. Also, the tips of the five claws could penetrate in to soil with small force requirement of BB-1.

The article "Biomimetic Rotary Tillage Blade Design for Reduced Torque and Energy Requirement" was published in 2021. Journal: Appl Bionics Biomech.

### 7.2. Effect of the Structure Characteristics of the Multiclaw Combination (GC-2) on the Torque of BB-1 in the Soil-Cutting Process

The rotary tillage blade started to break the soil after the whole body of the blade entered the soil, and then, soil wedge was formed in front of the blade as shown in Figure 15. Based on the previous study [20], the soil rupture distance ratio of the five-claw combination was about 19.6% smaller than the predicted values of simple blades. It indicated that the soil failure wedge of the BB-1 was significantly diminished so that a lower force was needed for soil shearing.  Figure 15(c) illustrated the difference in the soil failure wedges formed by CB and BB-1 separately. By the comparison of the soil failure wedges, it confirmed that the five claw structure could change the soil failure pattern of the rotary tiller blade to form a smaller soil failure wedge for minimizing the torque requirement largely.

In sum, BB-1 firstly enhanced the penetrating and sliding cutting performance of the cutting edge based on the GC-1 of the five claw tips and secondly diminished the soil failure wedge in the soil-cutting process based on the GC-2 of the multiclaw combination, thus largely reducing the torque of BB-1. The smaller torque requirement made BB-1 more efficient. Therefore, the GC of five fore claws of mole rats is more applicable to the geometric optimization of rotary tillage blades.

## 8. Conclusion

Biomimetic rotary tillage blades were designed to reduce the torque requirement according to the geometric characteristics (GC) of the five fore claws of mole rats, including the contour curves of the five claw tips (GC-1) and the structural characteristic of the multiclaw combination (GC-2). Results of soil bin tests and field experiments showed the following:

1. The order of influence on the torque was as follows: the rotary speed (*n*), the ratio of claw width to interval (*r*), and the inclined angle (*θ*), all of which have obvious impacts by further analyzing regression curves of the submodels and their corresponding derivation curves of factors. Moreover, for the purpose of the reduction in torque requirement of the rotary tiller blade, the optimal working combination was set by the response surface methodology: *r* = 1.25, *θ* = 60°, and *n* = 240 rpm
2. The new optimal biomimetic blade (BB-1) in this study and the reported optimal biomimetic (BB-2) of the literature [10] averagely reduced the torque requirement by 13.99% and 3.74%, respectively, compared with the conventional blade (CB)
3. Field comparison experiments also showed that the torques of BB-1 were averagely 17.00%, 16.88%, and 21.80% lower than those of CB at different rotary speeds, forward velocities, and tillage depths, respectively

Overall, the geometric structure of the five claws of mole rats may play an important role in reducing the torque and energy requirement of rotary tillage blades. This research also provides a new method to design other soil-engaging tools for achieving a minimum soil resistance and energy consumption.

The article "Biomimetic Rotary Tillage Blade Design for Reduced Torque and Energy Requirement" was published in 2021. Journal: Appl Bionics Biomech.

## Figures and Tables

**Figure 1:** (a) Motion diagram of the mole claws according to Scott and Richardson [16]. (b) Motion diagram of the rotary tillage blade.

**Figure 2:** (a) A mole rat and (b) the five fore claws.

**Figure 3:** The point clouds and contour curves of the five claws of the mole rat.

**Figure 4:** The fitting curves of the five claw tips of mole rats.

**Figure 5:** Configurations of rotary tillage blades: (a) the conventional; (b) the biomimetic.

**Figure 6:** Soil bin tests: (a) soil bin and test equipment and (b) test toolbar: 1: soil bin trolley; 2: torque sensor; 3: universal joint coupling; 4: gear box; 5: synchronous belt wheel; 6: rotary tillage blade; 7: rotary shaft; 8: blade holder.

**Figure 7:** Scheme of three sections in the soil bin.

**Figure 8:** Nine biomimetic rotary tillage blades designed for the soil bin tests.

**Figure 9:** Three types of the blades used in the comparative test: (a) CB; (b) BB-2; (c) BB-1.

**Figure 10:** (a) Equipment used in the field experiment; (b) sensor testing system.

**Figure 11:** (a) Regression curves of the submodels and (b) the derivation curves of factors.

**Figure 12:** Response surface diagrams of torque: (a) *n* = 240; (b) *θ* = 60°; (c) *r* = 1.50.

**Figure 13:** The torques of the three rotary tillage blades affected by rotary speed.

The article "Biomimetic Rotary Tillage Blade Design for Reduced Torque and Energy Requirement" was published in 2021. Journal: Appl Bionics Biomech.

**Figure 14:** Torques of rotary tiller blades at different tillage conditions: (a) rotary speed; (b) forward velocity; (c) tillage depth.

**Figure 15:** Soil wedge formed in front of the rotary tillage blade: (a) the conventional (CB); (b) the optimal biomimetic (BB-1); (c) the comparison between the CB and the BB-1. Note: ABEF—soil surface cut by the blade; CDEF—previously soil surface cut by the preceding blade; ABI1J1G1H1—soil wedge formed in front of the CB; ABI2J2G2H2—soil wedge formed in front of the BB-1.

**Figure 16:** The curvature analysis of the fitting curves of the five claw tips: (a) the 1st; (b) the 2nd; (c) the 3rd; (d) the 4th; (e) the 5th.

**Table 1:** Coefficients of fitting equations of the five claw tips.

Coefficient of equation	Claw				
	1st	2nd	3rd	4th	5th
*a*_1_	1.932	4.251	8.196	0.5015	1.657
*b*_1_	-0.6218	-0.7791	-0.6644	0.6707	0.5445
*c*_1_	0.7628	0.864	1.569	0.4673	0.5248
*a*_2_	5.789	5.658	5.318	3.937	2.473
*b*_2_	0.4466	0.6178	1.061	-0.1576	-0.2982
*c*_2_	1.563	1.178	1.165	1.673	0.7749
SSE	0.03953	0.01268	0.006721	0.003073	0.001469
*R* ^2^	0.9965	0.9803	0.9986	0.9975	0.9985
Adjusted *R*^2^	0.9959	0.9738	0.9983	0.9968	0.998
RMSE	0.03899	0.02907	0.01789	0.01272	0.009897

**Table 2:** Geometrical parameters and structural elements of the multiclaw combination.

Claw	*L* (mm)	*W* (mm)	$q=\frac{\;L}{W}$	Adjacent claws	Δ*x* (mm)	$r=\frac{\;\Delta x}{W}$
1^st^	6.47	2.34	2.76	1^st^ and 2^nd^	3.86	1.60
2^nd^	7.83	2.42	3.24	2^nd^ and 3^rd^	2.89	1.12
3^rd^	8.82	2.59	3.41	3^rd^ and 4^th^	3.04	1.17
4^th^	7.99	2.46	3.25	4^th^ and 5^th^	3.22	1.31
5^th^	5.43	2.06	2.63			

**Table 3:** Factor-level coding.

Factor	Code	Level		
		-1	0	1
*r*	*x*_1_	1.25	1.50	1.75
*θ* (°)	*x*_2_	50°	60°	70°
*n* (rpm)	*x*_3_	160	240	320

**Table 4:** Test scheme and result of coded test.

Number	*r*	*θ* (°)	*n* (rpm)	*x*_1_	*x*_2_	*x*_3_	*T* (N-m)
1	1.25	60°	160	-1	0	-1	23.84
2	1.50	60°	240	0	0	0	18.27
3	1.25	70°	240	-1	1	0	17.55
4	1.25	50°	240	-1	-1	0	17.26
5	1.50	70°	320	0	1	1	22.31
6	1.25	60°	320	-1	0	1	20.56
7	1.50	60°	240	0	0	0	18.33
8	1.75	50°	240	1	-1	0	19.05
9	1.75	60°	160	1	0	-1	25.81
10	1.50	50°	320	0	-1	1	22.06
11	1.50	60°	240	0	0	0	18.21
12	1.75	70°	240	1	1	0	19.33
13	1.50	60°	240	0	0	0	18.44
14	1.50	50°	160	0	-1	-1	24.85
15	1.50	70°	160	0	1	-1	25.51
16	1.50	60°	240	0	0	0	18.31
17	1.75	60°	320	1	0	1	22.58

**Table 5:** ANOVA table for the regression model.

Source of variation	Quadratic sum	Degree of freedom	Mean sum of square	*F*	*P*
Model	139.12	9	15.46	1090.96	<0.0001
*x*_1_	7.14	1	7.14	504.23	<0.0001
*x*_2_	0.27	1	0.27	19.32	0.0032
*x*_3_	19.53	1	19.53	1378.49	<0.0001
*x*_1_ *x*_2_	2.50*E* − 5	1	2.50*E* − 5	1.76*E* − 3	0.9677
*x*_1_ *x*_3_	6.25*E* − 4	1	6.25*E* − 4	0.044	0.8396
*x*_2_ *x*_3_	0.042	1	0.042	2.97	0.1287
*x*_1_ *x*_1_	0.26	1	0.26	18.54	0.0035
*x*_2_ *x*_2_	0.23	1	0.23	16.45	0.0048
*x*_3_ *x*_3_	111.03	1	111.03	7836.71	<0.0001
Residual	0.099	7	0.014		
Lack of fit	0.07	3	0.023	3.25	0.1426
Pure error	0.029	4	7.22*E* − 3		
Cor. total	139.22	16			

The article "Biomimetic Rotary Tillage Blade Design for Reduced Torque and Energy Requirement" was published in 2021. Journal: Appl Bionics Biomech.

## Data Availability

The data used to support the findings of this study are available from the first author upon request.
